RETRACTED

# Facile, one-pot biosynthesis and characterization of iron, copper and silver nanoparticles using *Syzygium cumini* leaf extract: As an effective antimicrobial and aflatoxin B_1_ adsorption agents

**DOI:** 10.1371/journal.pone.0234964

**Published:** 2020-07-02

**Authors:** Muhammad Asif Asghar, Erum Zahir, Muhammad Arif Asghar, Javed Iqbal, Ahad Abdul Rehman

**Affiliations:** 1 Food and Feed Safety Laboratory, Food and Marine Resources Research Centre, PCSIR Laboratories Complex, Shahrah-e-Salimuzzaman Siddiqui, Karachi, Pakistan; 2 Department of Chemistry, University of Karachi, Karachi, Pakistan; 3 Department of Pharmaceutics, Faculty of Pharmacy, Jinnah Sindh Medical University, Karachi, Pakistan; 4 Pharmaceutical Manufacturing Technology Centre, Bernal Institute, University of Limerick, Castletroy, Limerick, Ireland; 5 Department of Pharmacology, Faculty of Pharmacy, Jinnah Sindh Medical University, Karachi, Pakistan; Qatar University, QATAR

## Abstract

In this study, a facile, ecological and economical green method is described for the fabrication of iron (Fe), copper (Cu) and silver (Ag) nanoparticles (NPs) from the extract of *Syzygium cumini* leaves. The obtained metal NPs were categorized using UV/Vis, SEM, TEM, FTIR and EDX-ray spectroscopy techniques. The Fe-, Cu- and Ag-NPs were crystalline, spherical and size ranged from 40−52, 28−35 and 11−19 nm, respectively. The Ag-NPs showed excellent antimicrobial activities against methicillin- and vancomycin-resistance *Staphylococcus aureus* bacterial strains and *Aspergillus flavus* and *A*. *parasiticus* fungal species. Furthermore, the aflatoxins (AFs) production was also significantly inhibited when compared with the Fe- and Cu-NPs. In contrast, the adsorption results of NPs with aflatoxin B_1_ (AFB_1_) were observed as following order Fe->Cu->Ag-NPs. The Langmuir isotherm model well described the equilibrium data by the sorption capacity of Fe-NPs (105.3 ng mg^-1^), Cu-NPs (88.5 ng mg^-1^) and Ag-NPs (81.7 ng mg^-1^). The adsorption was found feasible, endothermic and follow the pseudo-second order kinetic model as revealed by the thermodynamic and kinetic studies. The present findings suggests that the green synthesis of metal NPs is a simple, sustainable, non-toxic, economical and energy-effective as compared to the others conventional approaches. In addition, synthesized metal NPs might be a promising AFs adsorbent for the detoxification of AFB_1_ in human and animal food/feed.

## Introduction

Apart from recent advancement, pathogenic moulds contamination associated in food and feed products are still major threat world-wide. The gram-positive bacteria *Staphylococcus aureus* is considered a historically and most frequently associated human pathogen and able to produce various diseases in human [1]. Furthermore, aflatoxins (AFs) contamination are considered one of the most hazardous toxins and commonly found in food and feed crops [2, 3]. AFs are derivative of difurocoumarin and produced by toxigenic species of *Aspergillus flavus* and *A*. *parasiticus*. To date, at least 20 different types of AFs such as aflatoxin B_1_, B_2_, G_1_ and G_2_ have been identified. However, aflatoxin B_1_ (AFB_1_) is considered one of the utmost potent carcinogens, hepatotoxic, mutagenic, immunosuppressive, neoplastic and teratogenic [4]. Various environmental elements such as agricultural practices, moisture, temperature, unseasonal rains, geographical location, storage and transportation are also favored the growth and production of *Aspergillus* and AFB_1_ contamination.

RETRACTED

The massive economic effects on the agriculture segment can also be considered because this contamination is able to decrease nutritional significance of food and feedstuff, reduction in meat production, reduced kidney and liver function, immune system suppression and finally created harmfulness to the consumers of dairy/ foodstuffs. So, numerous strategies have been recommended for the AFs detoxification from contaminated food and feedstuff [5–7]. Though, most of the reported methods are having certain drawbacks.

The one of the most effective method to adsorb AFB_1_ is the addition of non-nutritive adsorbent in the contaminated consumption that decreased the bioavailability of toxin in the gastrointestinal tract. However, the non-specificity and the higher cost are the major issues of these adsorbents. In addition, due to non-degradable property, cause deposited in environment when excreted in manure is another issue that restricted to use [8].

Currently, nanotechnology is emerging field with its applications in science and technology such as bioengineering and nanomedicines through targeted drug delivery for cancer therapy, biomedical applications, pharmaceutical industry, contrast agents in magnetic resonance imaging (MRI), biosensing and antibacterial and photocatalytic agent [9–16]. Nanoparticles (NPs) are using in some cosmetics, sunscreens, toothpaste, pharmaceutical and even in food products [17]. Metal NPs directly encounter with the human/ animal body, therefore, there is necessary to develop environmentally pleasant approaches for the synthesis of NPs without using of toxic or dangerous chemicals.

A variety of techniques have been reported for the NPs synthesis, which are too expensive, low compound conversions, high energy requirement or involved environmentally hazardous chemicals [18, 19]. Biosynthesis of metal NPs using different plants leaves extracts [14], roots [20], microorganisms like fungi [21] and bacteria [22] have been developed as a new method to improve or remove the above-mentioned physical and chemical approaches challenges. Amongst the numerous well-known approaches, plant-mediated green synthesis of NPs is considered a widely accepted technology recently. Green nanotechnology has become most popular over the chemical techniques as a facile, economical, environment-pleasant, readily scaled up, without high temperature, pressure and energy, biocompatible, without using toxic and redundant chemicals and safe for human therapeutic uses. Various plants leaves extracts such as *Gongronema Latifolium*, *Moringa oleifera*, bitter leave (*Veronica amygdalina)*, *Psidium guajava* have been utilized for the biosynthesis of metal NPs [23–26]. The flavonoids, phenolics, polysaccharides and terpenoids are the secondary metabolites present in the plant that are accountable primarily for the metal ions reduction into bulk metallic NPs preparation in the redox reaction to obtain nano-sized NPs that are non-toxic by transforming M^+^ to M^0^ and also act as a capping agent of the obtained NPs [25].

RETRACTED

So, in this study, iron, copper and silver NPs were prepared using *Syzygium cumini* leaves extract and characterized using different techniques. Furthermore, antibacterial, antifungal and adsorption of AFB_1_ properties of each NPs were assessed under various conditions. Additionally, the adsorption mechanism was also judged by the assessment of adsorption isotherm models, kinetic and thermodynamic parameters.

## Materials and methods

### Synthesis of metal nanoparticles

Ten grams chopped leaves were accurately weighed and boiled in the presence of 100 mL DI-H_2_O for 20 min at 80°C, cooled at room environment and filtered using Whatman filter paper no. 1. The solutions of FeCl_3_, CuSO_4_ and AgNO_3_ (0.010 mol/L) was separately added to the plant extract in the ratio of 1:1, 4:1 and 9:1 by volume, respectively. All mixtures were stirred and NPs were obtained through centrifugation for 10 min at 10,000 rpm. The solid masses were then separately rinsed with DI-H_2_O in triplicate to eliminate boundless biological particles followed by drying at 80°C for 3 hours in a vacuum oven.

### Characterization of metal nanoparticles

The confirmation of the NPs formation was assessed by the changes in color of reaction suspension. However, pH of the originator/ reducing agents before and after mixing was also used as another indicator. UV–Vis absorption spectrum of individual NPs were recorded using double beam spectrophotometer (Model no. UV-1700, Shimadzu, Japan) between 200–800 nm. The size distribution and surface morphology of each NPs were analyzed using SEM (Model # JEOL- JSM 6380A, Japan) and TEM measurements (Model # JEOL JEM-2100F, Japan) operating at 160 kV with a point-to-point resolution of 1.9 Å. EDX spectroscopy of the synthesized NPs was assessed for the confirmation of elemental composition using the SEM with EDX detector (Model # EX-54175jMU, Jeol Japan). FTIR spectra for the evaluation of functional groups were obtained in the range of 500−4000 cm^-1^ using Perkin-Elmer 100 spectrometer (Perkin-Elmer Inc, Waltham, MA) by the potassium bromide pellet (FTIR grade).

RETRACTED

### Antibacterial assay

The antibacterial property of each NPs was assessed against gram-positive methicillin- (MRSA) and vancomycin-resistance (VRSA) *Staphylococcus aureus* infectious strains using modified Oxford cup diffusion inhibition assays [27]. In brief, the new culture was prepared in the concentration of 0.2 OD_600_ containing 10^6^ colony-forming units (CFU) per mL. The diluted culture was spread on petri plates containing 1.5% w v^-1^ nutrient agar using a disinfected glass rod spreader. Then, sterilized Oxford cups (6 mm) were placed on the upper of nutrient agar, dispensed 50 μL of 1 mg mL^-1^ (50 μg) of each NPs suspension into each Oxford cup and kept at 37°C for 24 h. The activity was recorded by the formation of inhibition zone (mm) round the Oxford cup by calliper. Antibiotics, Vancomycin and Cefoxitin (30 μg disc^-1^) (Oxoid, UK) were considered as a control. Each study was obtained in triplicate and results are stated as average ± SEM.

#### Minimum inhibitory concentration (MIC)

Dilution broth method was utilized to evaluate the MIC for each metal NPs. In brief, each NPs in a concentration between 1‒512 μg mL^-1^ was prepared in 10 mL 0.8% (w v^-1^) nutrient broth medium separately and sterilized for 15 min at 121°C using Rexall autoclave (Kaohsiung, Taiwan). An aliquot of 25 μL comprising bacterial strains (10^6^ CFU mL^-1^) was dispensed in each concentration and incubated overnight under rotation at 120 rpm and 37 ± 2°C. After incubation time, an aliquot of 200 μL was transported into sterilized ELISA plates (96-well) and optical densities (ODs) were noted using an ELISA reader (Infinite 200; Tecan Systems, USA) at 600 nm. However, positive control with only NPs and negative control with only inoculums were too executed. Each trial was done in triplicate and described as average ± SD.

### Antifungal assay

The antifungal property of NPs was carried out against toxigenic strains of *Aspergillus flavus* and *A*. *parasiticus* and the production of aflatoxin (AFs) contamination [28]. Briefly, separately metal NPs in the amount of 10, 25, 50, 100 μg mL^-1^ were added into the separate flask containing 100 mL of Czapek Dox Liquid medium. All flasks were autoclaved for 15 min at 121°C and then let to cool at room temperature. An aliquot 1 mL (about 10^6^ spores mL^-1^) of pathogenic *Aspergillus* was introduced into each flask. The same protocols were applied for each kind of toxigenic strain (*A*. *flavus* and *A*. *parasiticus*). The positive control with alone spore suspension whereas negative control with only NPs were also tested with the mean time. Then, mixtures were retained for 15 days at 25 ± 2°C. The mixture was blended for 2 min at 5000 rpm and purified using Whatman filter paper. The filtrates were utilized to determine the level of AFs by HPLC as described underneath.

RETRACTED

#### Determination of AFs using HPLC

The AFs levels were determined using our previously described technique [2]. In short, AFs was extracted in triplicate with 50 mL of chloroform from culture filtrates. The chloroform extract was collected and evaporated in a rotary flask evaporator. The residue of each chloroform extract was re-suspended in 100 mL of methanol:water: (80:20; v v^-1^) and purified using Whatman filter paper. Two mL filtrate diluted with PBS (pH 7.4) was passed through AflaStar^TM^ immunoaffinity column (IACs). The column was washed two times with 20 mL of DI-H_2_O. The elution of AFs was done by passing 1.5 mL of HPLC grade methanol and DI-H_2_O in an amber vial. AFs were examined using HPLC attached with fluorescence sensor and post-column (Kobra Cell) derivatization. The mobile phase preparation was H_2_O:ACN:MeOH (65:17.5:17.5; v v^-1^) with KBr (119 mg L^-1^) and HNO_3_ (154 ml L^-1^) and delivered at 1 mL min^-1^. A volume of 99 μL of samples was introduced and separated using a LiChroCART^®^ 100Å RP-18 column (40°C).

### Adsorption of aflatoxin B_1_

The adsorption of aflatoxin B_1_ (AFB_1_) with each NPs was studied according to the previously defined method with some modifications [29]. NPs with the amount of 0.1−5 mg mL^-1^ were introduced separately in Erlenmeyer containers comprising AFB_1_ solution (100 ng mL^-1^) to examine the optimal NPs amount on which greater adsorption occurred. All flasks were placed in thermo shaker incubator for 45 min at 120 rpm at 37 ± 2°C. After a specific time period, centrifugation was performed for 2 min at 10,000 rpm. The supernatant was attained and free AFB_1_ was determined by HPLC as described above. The adsorption amount of AFB_1_ was obtained by the comparison of initial and equilibrium AFB_1_ concentrations in solution (***Eq 1***).

$$Adsorption\;(\%)=\frac{Ci-Ce}{Ci}\times 100$$ Eq (1)

*Where*, Ci / Ce (ng mL^-1^) are the initial / equilibrium AFB_1_ concentrations in solution respectively. The entire procedure was validated using the positive and negative controls.

RETRACTED

The adsorption experiments were performed with each NPs equivalent to 1 mg mL^-1^ and different initial concentrations of AFB_1_ solutions (20–200 ng mL^-1^). To reveal the release efficiency directly and adsorption isotherm, the adsorption experiments were performed with the constant amount of each NPs (1 mg mL^-1^) and different initial concentrations of AFB_1_ solutions (20–200 ng mL^-1^). The solutions were agitated in thermo shaker at 120 rpm and 37°C for 45 min. The AFB_1_ amount was determined by HPLC at equilibrium and time *t* = 0. Entirely trials were executed in triplicate and the AFB_1_ amount at equilibrium Qe (ng mg^-1^) was obtained by mass balance equation (***Eq 2***):

$$Qe=\frac{Ci-Ce}{M}\times V$$ Eq (2)

where

M (mg mL^-1^) and V (mL) are the amount and volume of NPs, respectively. The influence of pH was performed at initial pH of 1, 3, 5, 7 and 9. However, further factors were kept constant (37 ± 2°C, 45 min, NPs amount 1 mg and 100 ng mL^-1^ of AFB_1_ concentration). The kinetic study was evaluated as same with the equilibrium execution to investigate the effect of contact time. The solutions were composed by centrifugation after 15 min interval vigorous mixing. On regular time intervals, the AFB_1_concentrations in the supernatant was assessed at time t = 0 and t by HPLC. The temperature effect and thermodynamic parameters were estimated by incubation the samples at 10, 25, 37 and 45°C. The supernatant was utilized for the analysis of un-attached AFB_1_ by HPLC procedure. Entirely trials were carried out in three times.

## Results and discussion

### Formation and characterization of metal nanoparticles

The color variations from pale yellow to brownish black were the first indication for the formation of NPs. The further confirmation was done by the variation in the solutions pH. The mixture pH was tested pre- and post-reduction as mentioned in **Table 1**. Before and after reduction, the pH was observed as acidic. Though, the pH of the solution further decreased in the reduction route and moved to the more acidic range.

**Table 1:** Morphology and particles size distribution of metal NPs produced by *Syzygium cumini* (Jamun) leaves extract.

Nanoparticles IDs	Change in color		change in pH		Final yield (mg)	Morphology	Size (nm) Range (Mean)	
	Plant extract	After reduction	Plant extract	After reduction			SEM	TEM
Fe-NPs	Pale Yellow	Brownish Black	5.86	3.25	52.2	Spherical	40−52 (46)	30−42 (40)
Cu-NPs		Brown		3.36	36.9	Spherical	28−35 (31)	20−35 (30)
Ag-NPs		Brown		4.21	18.5	Spherical	11−19 (15)	7−14 (10)

NPs = nanoparticles, SEM = scanning electron microscope, TEM = Transmission Electron Microscopy

The SEM micrographs displayed that prepared NPs were agglomerated and spherical in nature **(Fig 1A–1C).** The diameter of Fe-, Cu- and Ag-NPs ranged (average) from 55−65 (58)-, 42−52 (45)- and 22−38 (32) nm, respectively **(Table 1)**. The difference in size was due to the different volume of leaves extract was used for the metal ions reduction. Consequently, the volume of leaves extract directly effects on the morphology, size and production of NPs. The presence of higher amount of polyphenols in the *Syzgium cumini* was the main reason for the larger size particles formation as reported by Kumar et al., (2010), as observed in the larger-sized Fe-NPs, where a lot of polyphenols present [30].

RETRACTED

**Fig 1:** SEM images of metal nanoparticles (a) iron (b) copper and (c) silver nanoparticles.

The TEM images of synthesized metal NPs **(Fig 2A–2C)** showed that a large number of NPs were in spherical form. The images revealed that the most of the NPs were agglomerated, due to hydroxyl arrangement of extract. Fe-, Cu- and Ag-NPs was observed to be around 40-, 30- and 10 nm in size, respectively **(Table 1)**, which is comparable with the NPs size as obtained from SEM results.

**Fig 2:** TEM images of metals nanoparticles (a) iron (b) copper and (c) silver nanoparticles.

The FTIR spectrum **(Fig 3A)** showed the incidence of various biomolecules such as flavonoids and polyphenols in *Syzgium cumini* leaves extract and able to produce NPs. The peak seemed at 1065 cm^-1^, which linked to C-N aliphatic amines stretching vibration or alcohols/ phenols. The sorption peak appears at 3425 cm^-1^ specifies polyphenolic OH molecule. The peak at about 3000 cm^-1^ corresponded with aromatic C-H broadening. At 3258 cm^-1^ peak can be attributed to primary aliphatic amines. The peaks appeared at 1620 and 1065 cm^-1^ shows the existence of carbonyl groups (C = O) and C-O single bonds, respectively. The aromatic C-H out of plane deformation bands found at 614 cm^-1^ [31]. **Fig 3B** displays the FTIR spectrum of Fe-NPs. The peaks detected at 3442 and 2924 cm^-1^ specifies to O−H broadening vibrations of the C−OH or H_2_O and CH_2_ stretching vibrations, respectively. However, the peaks at 1649 and 1091 cm^-1^ seems to be C = C and C-O particular bonds, respectively. The C−O−C of carboxylic acid exist at the boundaries of Fe-NPs appeared at 790 cm^-1^ [32]. At 569 cm^-1^ peak was appeared owing to Fe–O strecting [33]. **Fig 3C** presented the Cu-NPs FTIR spectrum which indicated the broad peaks at 3425 cm^-1^ and 1622 cm^-1^ associated to O–H groups and un-reacted ketone group indicating the existence of flavonones which adsorbed on the Cu-NPs surface, respectively. The peaks at 1471 and 1394 cm^-1^ indicated the polyphenolic O–H bend, verify the existence of aromatic cluster. The peak at 1111 cm^-1^ was allotted to C–O–C group in Cu-NPs [34]. The characteristic spectrum of synthesized Ag-NPs presented three bands among 823 and 1384 cm^-1^ **(Fig 3D)**. A broad band also appears at about 3412 cm^-1^ may be attributed to O−H and representing the promising participation in the NPs synthesis. However, two less intense and narrower bands appear between 1710 and 2385 cm^-1^. The peak at 1641 cm^-1^ is labelled to the C = O broadening vibration of acid derivatives. The peaks at 1381 cm^-1^ corresponding to C = C of amide groups and aromatic rings. The peak at 1070 cm^-1^ agrees to aliphatic amines C**−**N stretching vibration confirms the incidence of polyphenols [30].

RETRACTED

**Fig 3:** FTIR spectra of *Syzygium cumini* leaves extract and metal nanoparticles (a) *Syzygium cumini* leaves extract (b) iron (c) copper and (d) silver nanoparticles.

**Fig 4A** presented the EDX spectrum of Fe-NPs contains peaks of Fe, O and C in addition Na and Cl and C confirming the formation of Fe. The Cl signals must be resulting from FeCl_3_ precursors used in NPs formation. The EDX spectrum of Cu-NPs is presented in **Fig 4B**, indicates the C, O, S and Cu peaks. The peak of S obtained from CuSO_4_ precursors used in the synthesis protocol. The EDX profile of Ag-NPs showed in **Fig 4C**, a strong Ag signal in conjunction with Cl, C and O peaks, which may have created from the biomolecules present on the Ag-NPs surface.

**Fig 4:** EDX spectra of metal nanoparticles (a) iron (b) copper and (c) silver nanoparticles.

The optical property of synthesized Fe-, Cu- and Ag-NPs was assessed by the evaluation of UV-Vis spectra. Before the mixing of FeCl_3_, CuSO_4_ or AgNO_3_ solutions, the mustard or yellow colour of each plant extract don’t produces spectral features in UV/Vis range due to unavailability of surface plasmon resonance (SPR). However increasing in the absorbance after addition of precursor solutions indicated the onset of particles formation. UV-Vis spectrum of Fe-NPs revealed characteristic SPR absorption peak at 262 nm **(Fig 5A)** and agreement with the previous study [35]. UV/Vis spectrum of Cu-NPs presented maximum SPR absorption peak at 572 nm (**Fig 5B**). The strong SPR absorption band might be due to the SPR band of Cu colloids and the formation of NPs [36]. UV/Vis spectrum of Ag-NPs showed characteristic SPR absorption peak at 426 nm (**Fig 5C**), as compare with the previous study [23]. The increases in SPR absorption peak with respect to time indicating polydispersity nature of the Ag-NPs [37]. Only one sharp peak appeared in all spectrums, can be attributed to the NPs absorption and validates the NPs formation only. This phenomenon was occurred due to the SPR absorption and confirms that the protein of plant leaves act as a template and stabilizing agent during the synthesis of NPs. SPR is an important optical biosensing tool that occurs due to the combined vibration of electrons of metal NPs in resonance with the light wave.

RETRACTED

**Fig 5:** UV-Visible spectra of metal nanoparticles (a) iron (b) copper and (c) silver nanoparticles.

### Antibacterial study of metal nanoparticles

The zone of inhibition (ZOI) produced by NPs against MRSA and VRSA is presented in **Fig 6A and 6B**. However, the values of ZOI and MIC are presented in **Table 2**. The order of antibacterial property was found to be Ag- > Cu- > Fe-NPs, which shows that the NPs size is the important factor in the effect of antibacterial activity. It was clear from SEM and TEM studies that the size of Ag-NPs was smaller as compared with Cu- and Fe-NPs. The antibacterial effect of each NPs was considerably dissimilar with each other at *p ≤ 0*.*05*.

**Fig 6:** Zone of inhibition of produced by iron, copper and silver nanoparticles against *Staphylococcus aureus* strains (a) MRSA and (b) VRSA.

**Table 2:** The values of inhibition zone and minimum inhibitory concentration (MIC) of Fe-, Cu- and Ag-NPs against methicillin-resistance and vancomycin-resistance *Staphylococcus Aureus*.

NPs IDs	MRSA		VRSA	
	Zone of inhibition (mm ± SEM)	MIC ± SD (μg mL^-1^)	Zone of inhibition (mm ± SEM)	MIC ± SD (μg mL^-1^)
Fe-NPs	11 ± 0.45	128 ± 1.8	13 ± 0.28	128 ± 2.1
Cu-NPs	14 ± 0.33	32 ± 1.1	16 ± 0.31	32 ± 0.9
Ag-NPs	18 ± 0.32	8 ± 0.40	20 ± 0.40	8 ± 0.27

NPS = nanoparticles, SEM = standard error mean, SD = standard deviation.

The antibacterial activity of each NPs was considerably dissimilar from each other at *p ≤ 0*.*05*.

The greater surface area is provided by the smaller size of Ag-NPs, which delivers better contact to the microorganisms and showed superior antibacterial activity. Furthermore, Ag-NPs with small size comprises easier uptake, greater external area and as a results provides the efficiency in preventing the bacterial growth [38]. The MIC rate of Ag-NPs existed 4 and 8 times greater as related with Cu- and Fe-NPs, respectively. Whereas, the Cu-NPs shown 4 times additional bactericidal effect as Fe-NPs against MRSA / VRSA **(Table 2)**.

Various mechanisms have been proposed to understand the antibacterial performance of NPs. Oxidative stress caused by reactive oxygen species (ROS) is considered the key mechanism by which these particles showed antibacterial activity. NPs can generate ROS that is responsible for damaging the proteins and DNA of bacteria’s cells and finally death. This is the main mechanism by which antibacterial drugs and antibiotics work [38]. Furthermore, the NPs connect to the cell membrane of microbes and penetrated in to the cell. NPs interconnect with the phosphorus-comprising compounds such as DNA and sulfur-holding proteins, resulting in the distortion of helical arrangements and interferes essential biochemical reactions. A small molecular load area in the bacteria center is produced by NPs, consequently, protecting the DNA with the metal ions. NPs may hit the respiratory circle, blocked the cell partition finally leading to cell decease [39].

RETRACTED

### Antifungal study of metal nanoparticles

The antifungal action of NPs was in the increasing order Fe- < Cu- < Ag-NPs and associated with the dose of particles **(Table 3)**. Ag-NPs presented a strong antifungal effect in contradiction of *Aspergillus* species and inhibit the production of aflatoxins (AFs). For instance, no AFs (100% inhibition) was produced at 100 μg mL^-1^ of Ag-NPs in both strains. However, about 43−49% and 76−80% reduction was achieved using Fe- and Cu-NPs, respectively. The antifungal effect of individually NPs was considerably dissimilar with each other at *p ≤ 0*.*05*. As mentioned above, the smaller size NPs have significantly antibacterial/ antifungal activity as compare to the larger particles. The greater antimicrobial effect of Ag-NPs can be correlated with their size and shape which provides greater surface area [38]. Venkatesan et al., (2016) also described the superior antifungal effect of Ag-NPs amongst other NPs and commercially accessible antifungal agents, as agree with this study [40]. The inhibition rate was increased by the increased amount of NPs.

**Table 3:** Influence of various amounts of Fe-, Cu- and Ag-NPs on aflatoxins contamination produced by *Aspergillus flavus* and *A*. *parasiticus*.

Amount of nanoparticles (μg mL^-1^)	Reduction (%) of aflatoxins at different amount of Fe-, Cu- and Ag-NPs					
	*Aspergillus flavus*			*Aspergillus parasiticus*		
	Fe-NPs	Cu-NPs	Ag-NPs	Fe-NPs	Cu-NPs	Ag-NPs
10	3.4 ± 0.4	9.9 ± 1.2	35.8 ± 2.2	4.1 ± 0.4	15.2 ± 1.9	38.6 ± 2.7
25	9.1 ± 1.9	25.8 ± 1.8	48.1 ± 3.2	11.5 ± 1.4	32.5 ± 1.6	53.6 ± 3.0
50	25.6 ± 1.3	47.8 ± 2.2	66.4 ± 2.8	30.3 ± 1.5	55.8 ± 3.2	69.7 ± 3.1
100	43.9 ± 1.4	75.7 ± 3.2	100 ± 0.0	49.0 ± 1.8	80.0 ± 2.1	100 ± 0.0

The antifungal activity of each NPs was considerably dissimilar from each other at *p ≤ 0*.*05*.

Different reports are available in which the antifungal mechanism of NPs was described. The best mechanism in which NPs is joined with the cell wall and move inside the cell. NPs interrelate with protein and DNA and generate mutation process. As a result, DNA not capable to reproduce and stop the cell partition finally in cell decease [41]. Furthermore, NPs are able to create a spot of low molecular area at the midpoint of fungi cell. The particles then disrupt the respiratory arrangement and eventually cell splitting is entirely stopped subsequent in cell death [42]. The damage and rupture cell membrane can also be seen in the SEM micrograph after the treated with NPs and lastly cell death [28].

RETRACTED

### Adsorption of aflatoxin B_1_

In the present study, the adsorption ability of NPs with AFB_1_ was optimized by altering the amount of NPs, AFB_1_ concentration, pH, incubation temperature and time.

#### Effect of nanoparticles amount

**Fig 7A** provides the outcome of NPs quantity on the adsorption route, which indicates that the rate of AFB_1_ adsorption improved with increasing amount of NPs. When the amount of adsorbent rises, the sorption places on the surface of adsorbent was also increases, consequently increasing the AFB_1_ adsorption rate [43]. The adsorption ability of individually NPs was also likened; it was noticed that Fe-NPs having greater adsorption ability with AFB_1_ than Cu- and Ag-NPs.

**Fig 7:** Effect of different parameters on the adsorption of aflatoxin B_1_ using iron, copper and silver nanoparticles (a) Effect of nanoparticles amount (b) Effect of initial concentration of aflatoxin B_1_ (c) Effect of pH (d) Effect of incubation time and (e) Effect of incubation temperature. Blue Iron nanoparticles red copper nanoparticles green silver nanoparticles.

#### Effect of aflatoxin B_1_ concentration

The influence of AFB_1_ concentration on the sorption method is presented in **Fig 7B**. The adsorption of AFB_1_ declined with increasing the primary concentration of AFB_1_. At the higher AFB_1_ concentration, the adsorption positions of NPs completely saturated. The adsorption sites were completely engaged and vacancies for adsorption were not available. Consequently, a gradual decline was documented in the sorption amount.

#### Effect of pH

The adsorption ability of NPs with respect to pH is shown in **Fig 7C**, that adsorption of AFB_1_ continuously increases with arise in solution pH. At lower pH, more positive charges (H^+^) exist on the NPs surface, which provide large electrostatic repulsion strength between AFB_1_ and NPs. As pH increases, H^+^ ions can be certainly dissociated and the static repulsion forces drops and the AFB_1_ adsorption proliferations [44]. Furthermore, the charges and chemical interface among NPs and AFB_1_ are also contributed to this phenomenon. The pKa (constant of acid dissociation) is accountable for the AFB_1_charge [45].

RETRACTED

#### Effect of contact time

The AFB_1_adsorption with NPs was observed time-related and increases with increase in contact time (**Fig 7D**). The plot of AFB_1_ adsorption versus time presented that the rate of AFB_1_ adsorption was fast at the early periods and then extend progressively rises as the system achieved equilibrium. This suggests that the electrostatic attraction is the base of adsorption process [46]. The higher interval might be promoting the contact of ions to the adsorbent active sites; consequently, the maximum adsorption amount was attained. Moreover, the Fe-NPs provide higher adsorption degree than that of Cu- and Ag-NPs, that can be documented to its more interlamellar positioning that is promising to the distribution of AFB_1_ molecules [27].

#### Effect of incubation temperature

The adsorption ability of NPs was increased with rising the temperature (**Fig 7E**). This behavior indicates that the process was attained in endothermic nature. This may be due to increase AFB_1_ motility and creates or increases the number of active sites for the sorption procedure at greater temperature [47].

### Adsorption isotherm

The sorption mechanism was assessed by the calculation of three isotherm models such as Langmuir, Freundlich and Dubinin–Radushkevich (D-R) [48–50]. The fitness of isotherm model was done by the comparison of experimental and theoretical adsorption capacities (Qe) and regression correlation coefficient (R^2^) values. The isotherm parameters and R^2^ values are described in **Table 4**. The sorption data were well fixed by the Langmuir model. The experimental and theoretical Qe values are adjacent to each other with high R^2^ (0.970−0.979) values in contrast to Freundlich and D-R models. The Langmuir model describes the monolayer coverage on the NPs surface with AFB_1_. The phenomena occur due to the uniform spreading of active positions on the NPs edges.

**Table 4:** The correlation and equilibrium isotherm constants for the sorption of aflatoxin B_1_ with Fe-, Cu- and Ag-NPs.

Nanoparticles IDs	Qe (exp)	Langmuir				Freundlich			D-R		
		Qmax	b	R_L_	R^2^	KF	n	R^2^	Qmax	Es	R^2^
Fe-NPs	102.6	105.3	0.158	0.863	0.970	0.351	3.300	0.944	38.0	0.0263	0.923
CU-NPs	87.4	88.5	0.138	0.879	0.979	0.375	4.329	0.968	43.7	0.0229	0.907
Ag-NPs	80.0	81.7	0.115	0.897	0.979	0.324	4.054	0.971	39.1	0.0256	0.942

Qe = equilibrium concentration, Q_max_ = capacity of monolayer, b = Langmuir constant, R_L_ = separation constant factor, R^2^ = determination coefficients, K_F_ = sorption capacity, n = sorption intensity, Es = mean free energy of adsorption, DR = Dubinin–Radushkevich adsorption isotherm.

RETRACTED

The Q_max_ values of each NPs was considerably dissimilar each other at *p ≤ 0*.*05*.

The maximum Qe values of Fe-, Cu- and Ag-NPs with AFB_1_ were 105.3-, 88.5- and 81.7 ng mg^-1^, respectively. Furthermore, the R_L_ values of Langmuir constant were found > 0 but < 1, showing that the process was quite favorable and other contents is not affected the process. In addition, the values of Es were estimated by D-R model were between 0.0407−0.0439 kJ mol^-1^, indicating inside the physical adsorption energy range equivalent to 8 kJ mol^-1^ [51].

### Kinetic study

In order to examine the rate of sorption process of NPs with AFB_1_, pseudo-first and pseudo-second order kinetics models were applied. The selection of model existed on the values of experimental and theoretical Qe and R^2^. The kinetic parameters and R^2^ values are accessible in **Table 5**. The sorption data were well verifying the condition by the pseudo-second order kinetics model. The experimental and theoretical values of Qe were agreed to each with the linear plot (R^2^ close to 1). The data suggested that the environment of the process was a chemical monitoring procedure. Furthermore, the electrostatic interface among NPs and AFB_1_ could also be deliberated in the adsorption manner. The chemisorption is recognized as the rate limiting step and attributed the very fast kinetics to adsorbate being adsorbed onto the adsorbent surface [52]. The initial adsorption rate (*h*) values were found higher due to more mass transfer action from higher initial concentrations. However, the adsorption rate (*k*_2_) values designates that the higher AFB_1_concentration should have caused in more driving forces and quicker rates for AFB_1_. As a result, the structural arrangement of active sites or functional groups available on the NPs surface was more promising for the binding of AFB_1_ [27].

**Table 5:** Kinetic parameters for aflatoxins B_1_ adsorption on Fe-, Cu- and Ag-NPs.

Nanoparticles IDs	Qe (exp)	First Order			Second Order			
		R^2^	K_1_ (min^-1^)	Qe (Calc)	R^2^	K_2_ (min^-1^)	Qe (Calc)	h
GT-Fe-NPs	102.6	0.8390	0.1059	1.79	0.9920	0.0004	106.42	3.97
BT-Fe-NPs	87.4	0.7780	0.1105	1.82	0.9790	0.0005	90.91	3.86
GT-Cu-NPs	80.0	0.8730	0.0484	2.31	0.9860	0.0004	84.75	2.75

Qe = equilibrium concentration, R^2^ = determination coefficients, K_1_ = Lagergren (pseudo-first order) adsorption rate constant, K_2_ = pseudo-second order adsorption rate constant, h = initial sorption rate.

The Q_e_ values of each NPs was considerably dissimilar each other at *p ≤ 0*.*05*.

RETRACTED

### Thermodynamic parameters

The thermodynamic parameters such as Gibbs free energy (*ΔG°*), enthalpy (*ΔH°*), and entropy (*ΔS°*) of the AFB_1_ adsorption with NPs were determined using Van’t Hoff equation at different temperatures [53]. The obtained parameters are showing in **Table 6**. The *ΔG°* values of process were calculated negative for each tested temperatures, specified that the process was feasible, spontaneous and endothermic. Additionally, as the temperature rises the *ΔG°* values improved, proposing that the sorption may be more feasible at greater temperature. A similar pattern for the adsorption of AFB_1_ using grape pomace, banana peel and magnetic carbon nanocomposites obtained from bagasse have been studied and indicate that the adsorption process occurs spontaneously at a higher temperature [47, 54, 55]. The positive values of *ΔH°* showing the endothermic nature of adsorption process and improved the randomness of the solid-solution. The amount of the *ΔH°* values also offers indication of the environment of the adsorption, values < 20 kj mol^-1^ reflected indicative of physiosorption rather than chemisorptions. The *ΔH°* values determined for AFB_1_ on NPs ranged from 5.66 to 7.42 kj mol^-1^ suggesting physiosorption process and confirms the endothermic process. Whereas, the *ΔS°* values were also positive and higher for each NPs, which surmise that the adsorption process was favorable in terms of entropy. The *ΔS°* values also designated the increased randomness at the adsorbent/solution interface during the adsorption process [56].

**Table 6:** Thermodynamic considerations of the adsorption aflatoxins B_1_ with Fe-, Cu- and Ag-NPs.

Nanoparticles IDs	ΔH° (kJ mol^-1^)	ΔS° (J mol.K^-1^)	ΔG° (kJ mol^-1^) at different temperature (K)			
			298	303	308	313
Fe-NPs	7.42	34.17	-2.23	-2.86	-3.04	-3.52
Cu-NPs	6.70	29.67	-1.70	-2.14	-2.48	-2.75
Ag-NPs	5.66	23.77	-1.07	-1.42	-1.69	-1.91

K = Kelvin; ΔG° = Gibbs free energy; ΔH° = enthalpy; ΔS° = entropy

The ΔG°, ΔH° and ΔS° values of each NPs were considerably dissimilar at *p ≤ 0*.*05*.

## Conclusion

In this study, Fe-, Cu- and Ag-NPs were effectively produced using *Syzgium cumini* leaves extract. Ag-NPs display the more significant antimicrobial activity and reduced the production of AFs contamination as compare to Cu- and Fe-NPs. In addition, Fe-NPs showed the higher adsorption capacity with AFB_1_ in contrast to Cu- and Ag-NPs. In conclusion, metal NPs synthesized by *Syzgium cumini* leaves may be applied in biomedical uses, remedial in industrial purposes, the alternative of Cefoxitin and Vancomycin antibiotic and preparation of antimicrobial drugs. Metal NPs can also be apply as an active fungicide in the cultivated process, preparation of medicine and pesticide and controlling phytopathogenic microorganisms and AFs contamination. In addition, NPs can be used as an alternative of commercially available AFs adsorbent for the detoxification of AFB_1_ in human and animal food/ feed.

RETRACTED

## Supporting information

S1 Fig (PDF)

## References

[1] KaoCH, KuoYC, ChenCC, ChangYT, ChenYS, WannSR, et al Isolated pathogens and clinical outcomes of adult bacteremia in the emergency department: a retrospective study in a tertiary Referral Center. J Microbiol Immunol Infect. 2011;44:215–221.2152461710.1016/j.jmii.2011.01.023

[2] AsgharMA, AhmedA, ZahirE, AsgharMA, IqbalJ, WalkerG. Incidence of aflatoxins contamination in dry fruits and edible nuts collected from Pakistan. Food Cont. 2017;78:169–175.

[3] BrydenWL. Mycotoxins in the food chain: human health implications. Asia Pac J Clin Nutr. 2007;16:95–101.17392084

[4] AsgharMA, IqbalJ, AhmedA, KhanMA. Occurrence of aflatoxins contamination in brown rice from Pakistan. Iran J Public Health. 2014;43:291–299. 25988088PMC4419166

[5] MartinsLM, Sant'AnaAS, IamanakaBT, BertoMI, PittJI, TaniwakiMH. Kinetics of aflatoxin degradation during peanut roasting. Food Res Intern. 2017;97:178–183.10.1016/j.foodres.2017.03.05228578039

[6] MobeenA, AftabA, AsifA, ZuzzerA. Aflatoxins B1 and B2 contamination of peanut and peanut products and subsequent microwave detoxification. J Pharm Nutr Sci. 2011;1:1–3.

[7] TripathiS, MishraH. Studies on the efficacy of physical, chemical and biological aflatoxin B1 detoxification approaches in red chilli powder. Intern J Food Saf Nutr Public Health. 2009;2:69–77.

[8] HuwigA, FreimundS, KäppeliO, DutlerH. Mycotoxin detoxication of animal feed by different adsorbents. Toxicol Lett. 2001;122:179–188.1143922410.1016/s0378-4274(01)00360-5

[9] ParkJ, KadasalaNR, AbouelmagdSA, CastanaresMA, CollinsDS, WeiA, et al Polymer–iron oxide composite nanoparticles for EPR-independent drug delivery. Biomater. 2016;101:285–295.10.1016/j.biomaterials.2016.06.007PMC492129727310916

[10] AisidaSO, AkpaPA, AhmadI, ZhaoT-k, MaazaM, EzemaFI. Bio-inspired encapsulation and functionalization of iron oxide nanoparticles for biomedical applications. Eur Polym J. 2020;122:109371.

[11] KuppusamyP, YusoffMM, ManiamGP, GovindanN. Biosynthesis of metallic nanoparticles using plant derivatives and their new avenues in pharmacological applications–An updated report. Saudi Pharm J. 2016;24:473–484.2733037810.1016/j.jsps.2014.11.013PMC4908060

[12] LiY, LiCH, TalhamDR. One-step synthesis of gradient gadolinium ironhexacyanoferrate nanoparticles: a new particle design easily combining MRI contrast and photothermal therapy. Nanoscale. 2015;7:5209–5216.2570605710.1039/c4nr06481j

RETRACTED

[13] GeorgeJM, AntonyA, MathewB. Metal oxide nanoparticles in electrochemical sensing and biosensing: a review. Microchim Acta. 2018;185(7):358.10.1007/s00604-018-2894-329974265

[14] MadubuonuN, AisidaSO, AliA, AhmadI, ZhaoT-k, BothaS, et al Biosynthesis of iron oxide nanoparticles via a composite of Psidium guavaja-Moringa oleifera and their antibacterial and photocatalytic study. J Photochem Photobiol B: Biol. 2019;199:111601.10.1016/j.jphotobiol.2019.11160131470270

[15] UgwokeE, AisidaSO, MirbaharAA, ArshadM, AhmadI, ZhaoT-k, et al Concentration induced properties of silver nanoparticles and their antibacterial study. Surf Interfaces. 2020;18:100419.

[16] AisidaSO, UgwokeE, UwaisA, IroegbuC, BothaS, AhmadI, et al Incubation period induced biogenic synthesis of PEG enhanced Moringa oleifera silver nanocapsules and its antibacterial activity. J Polym Res. 2019;26:225.

[17] HoetPH, Brüske-HohlfeldI, SalataOV. Nanoparticles–known and unknown health risks. J Nanobiotechnol. 2004;2:12.10.1186/1477-3155-2-12PMC54457815588280

[18] IravaniS, KorbekandiH, MirmohammadiSV, ZolfaghariB. Synthesis of silver nanoparticles: chemical, physical and biological methods. Res Pharm Sci. 2014;9(6):385 26339255PMC4326978

[19] HasanpoorM, AliofkhazraeiM, DelavariH. Microwave-assisted synthesis of zinc oxide nanoparticles. Proced Mater Sci. 2015;11:320–325.

[20] BehravanM, PanahiAH, NaghizadehA, ZiaeeM, MahdaviR, MirzapourA. Facile green synthesis of silver nanoparticles using Berberis vulgaris leaf and root aqueous extract and its antibacterial activity. Int J Biol Macromol. 2019;124:148–154.3044736010.1016/j.ijbiomac.2018.11.101

[21] YadavA, KonK, KratosovaG, DuranN, IngleAP, RaiM. Fungi as an efficient mycosystem for the synthesis of metal nanoparticles: progress and key aspects of research. Biotechnol Lett. 2015;37:2099–2120.2616470210.1007/s10529-015-1901-6

[22] SalunkeBK, SawantSS, LeeS-I, KimBS. Microorganisms as efficient biosystem for the synthesis of metal nanoparticles: current scenario and future possibilities. World J Microb Biot. 2016;32:88.10.1007/s11274-016-2044-127038958

[23] AisidaSO, UgwuK, AkpaPA, NwanyaAC, EjikemePM, BothaS, et al Biogenic synthesis and antibacterial activity of controlled silver nanoparticles using an extract of Gongronema Latifolium. Mater Chem Phy. 2019;237:121859.

[24] AisidaSO, MadubuonuN, AlnasirMH, AhmadI, BothaS, MaazaM, et al Biogenic synthesis of iron oxide nanorods using Moringa oleifera leaf extract for antibacterial applications. Appl Nanosci. 2020;10:305–315.

[25] AisidaSO, UgwuK, AkpaPA, NwanyaAC, NwankwoU, BothaSS, et al Biosynthesis of silver nanoparticles using bitter leave (Veronica amygdalina) for antibacterial activities. Surf Interfaces. 2019;17:100359.

RETRACTED

[26] MadubuonuN, AisidaSO, AhmadI, BothaS, ZhaoT-k, MaazaM, et al Bio-inspired iron oxide nanoparticles using Psidium guajava aqueous extract for antibacterial activity. Appl Phy A. 2020;126(1):1–8.

[27] AsgharMA, ZahirE, ShahidSM, KhanMN, AsgharMA, IqbalJ, et al Iron, copper and silver nanoparticles: Green synthesis using green and black tea leaves extracts and evaluation of antibacterial, antifungal and aflatoxin B1 adsorption activity. LWT. 2018;90:98–107.

[28] HassanA, HowaydaM, MahmoudH. Effect of zinc oxide nanoparticles on the growth of mycotoxigenic mould. SCPT. 2013;1:66–74.

[29] AsgharM, IqbalJ, AhmedA, InamM, KhanM, JameelK. In vitro aflatoxins adsorption by silicon dioxide in naturally contaminated maize (Zea mays L.) and compared with activated charcoal. Res J Agri Biol Sci. 2015;11(3):9–16.

[30] KumarV, YadavSC, YadavSK. Syzygium cumini leaf and seed extract mediated biosynthesis of silver nanoparticles and their characterization. J Chem Tech Biot. 2010;85(10):1301–1309.

[31] BanerjeeJ, NarendhirakannanR. Biosynthesis of silver nanoparticles from Syzygium cumini (L.) seed extract and evaluation of their in vitro antioxidant activities. Dig J Nanomater Biostruct. 2011;6(3):961–968.

[32] MachadoS, PintoS, GrossoJ, NouwsH, AlbergariaJT, Delerue-MatosC. Green production of zero-valent iron nanoparticles using tree leaf extracts. Sci Total Environ. 2013;445:1–8.2329878810.1016/j.scitotenv.2012.12.033

[33] SunX, ZhengC, ZhangF, YangY, WuG, YuA, et al Size-controlled synthesis of magnetite (Fe3O4) nanoparticles coated with glucose and gluconic acid from a single Fe (III) precursor by a sucrose bifunctional hydrothermal method. J Phy Chem C. 2009;113(36):16002–16008.

[34] KeihanAH, VeisiH, VeasiH. Green synthesis and characterization of spherical copper nanoparticles as organometallic antibacterial agent. Appl Organomet Chem. 2017;31(7):e3642.

[35] NathD, ManharAK, GuptaK, SaikiaD, DasSK, MandalM. Phytosynthesized iron nanoparticles: effects on fermentative hydrogen production by Enterobacter cloacae DH-89. Bull Mater Sci. 2015;38(6):1533–1538.

[36] ZhangH-X, SiegertU, LiuR, CaiW-B. Facile fabrication of ultrafine copper nanoparticles in organic solvent. Nanoscale Res Lett. 2009;4(7):705–708. 10.1007/s11671-009-9301-2 20596465PMC2893818

[37] BeheraS, NayakP. In vitro antibacterial activity of green synthesized silver nanoparticles using jamun extract against multiple drug resistant bacteria. World J Nano Sci Tech. 2013;2(1):62–65.

[38] ReidyB, HaaseA, LuchA, DawsonKA, LynchI. Mechanisms of silver nanoparticle release, transformation and toxicity: a critical review of current knowledge and recommendations for future studies and applications. Mater. 2013;6(6):2295–2350.10.3390/ma6062295PMC545894328809275

RETRACTED

[39] BondarenkoO, IvaskA, KäkinenA, KurvetI, KahruA. Particle-cell contact enhances antibacterial activity of silver nanoparticles. PLoS One. 2013;8(5):e64060 10.1371/journal.pone.0064060 23737965PMC3667828

[40] VenkatesanJ, KimS-K, ShimMS. Antimicrobial, antioxidant, and anticancer activities of biosynthesized silver nanoparticles using marine algae Ecklonia cava. Nanomater. 2016;6(12):235.10.3390/nano6120235PMC530272428335363

[41] NasrollahiA, PourshamsianK, MansourkiaeeP. Antifungal activity of silver nanoparticles on some of fungi. Int J Nano Dimen. 2011;1:233–239.

[42] StoimenovPK, KlingerRL, MarchinGL, KlabundeKJ. Metal oxide nanoparticles as bactericidal agents. Langmuir. 2002;18(17):6679–6686.

[43] SallehMAM, MahmoudDK, KarimWAWA, IdrisA. Cationic and anionic dye adsorption by agricultural solid wastes: A comprehensive review. Desalin. 2011;280(1–3):1–13.

[44] YeS-Q, LvX-Z, ZhouA-G. In vitro evaluation of the efficacy of sodium humate as an aflatoxin B1 adsorbent. Aust J Basic Appl Sci. 2009;3(2):1296–1300.

[45] AvantaggiatoG, HavenaarR, ViscontiA. Assessment of the multi-mycotoxin-binding efficacy of a carbon/aluminosilicate-based product in an in vitro gastrointestinal model. J Agri Food Chem. 2007;55(12):4810–4819.10.1021/jf070280317511466

[46] SharZH, FletcherMT, SumbalGA, SheraziSTH, GilesC, BhangerMI, et al Banana peel: an effective biosorbent for aflatoxins Part A Chemistry, analysis, control, exposure & risk assessment. Food Addit Contam. 2016;33:849–860. 10.1080/0265203040000425927052947

[47] ZahoorM, KhanFA. Adsorption of aflatoxin B1 on magnetic carbon nanocomposites prepared from bagasse. Arab J Chem. 2018;11(5):729–738.

[48] LangmuirI. The constitution and fundamental properties of solids and liquids. Part I. Solids. J Am Chem Soc. 1916;38(11):2221–2295.

[49] FreundlichH. Over the adsorption in solution. J Phys Chem. 1906;57(385471):1100–1107.

[50] DubininM. The potential theory of adsorption of gases and vapors for adsorbents with energetically nonuniform surfaces. Chem Rev. 1960;60(2):235–241.

[51] GhadimEE, ManouchehriF, SoleimaniG, HosseiniH, KimiagarS, NafisiS. Adsorption properties of tetracycline onto graphene oxide: equilibrium, kinetic and thermodynamic studies. PLoS One. 2013;8(11):e79254 10.1371/journal.pone.0079254 24302989PMC3841164

[52] MayakaduwaS, KumarathilakaP, HerathI, AhmadM, Al-WabelM, OkYS, et al Equilibrium and kinetic mechanisms of woody biochar on aqueous glyphosate removal. Chemosphere. 2016;144:2516–2521. 10.1016/j.chemosphere.2015.07.080 26340852

RETRACTED

[53] SprynskyyM, Gadzała-KopciuchR, NowakK, BuszewskiB. Removal of zearalenone toxin from synthetics gastric and body fluids using talc and diatomite: A batch kinetic study. Colloids and Surf B: Biointerfaces. 2012;94:7–14.2232634010.1016/j.colsurfb.2011.12.024

[54] AvantaggiatoG, GrecoD, DamascelliA, SolfrizzoM, ViscontiA. Assessment of multi-mycotoxin adsorption efficacy of grape pomace. J Agri Food Chem. 2014;62(2):497–507.10.1021/jf404179h24364566

[55] SharZH, FletcherMT, SumbalGA, SheraziSTH, GilesC, BhangerMI, et al Banana peel: an effective biosorbent for aflatoxins. Food Addit Contam: Part A. 2016;33(5):849–860.10.1080/19440049.2016.117515527052947

[56] LiY, LiuT, DuQ, SunJ, XiaY, WangZ, et al Adsorption of cationic red X-GRL from aqueous solutions by graphene: equilibrium, kinetics and thermodynamics study. Chem Biochem Eng Q. 2011;25(4):483–491.

